The article "Caries-Preventive Effect and Retention of Glass-Ionomer and Resin-Based Sealants: A Randomized Clinical Comparative Evaluation" was published in 2022. Journal: Biomed Res Int.

# Caries-Preventive Effect and Retention of Glass-Ionomer and Resin-Based Sealants: A Randomized Clinical Comparative Evaluation

**DOI:** 10.1155/2022/7205692

**Published:** 2022-06-20

**Authors:** Ilhan Uzel, Ceren Gurlek, Berna Kuter, Fahinur Ertugrul, Ece Eden

**Affiliations:** ^1^Department of Pediatric Dentistry, Ege University, Izmir, Turkey; ^2^Bornova Oral and Dental Health Center, Izmir, Turkey; ^3^Izmir Demokrasi University, Faculty of Dentistry, Department of Pediatric Dentistry, Izmir, Turkey

## Abstract

**Background:**

Deep fissures are highly unprotected from the development of caries. Resin-based materials and glass-ionomer cements for sealing fissures are useful in caries control through physical barrier formation, which prohibits metabolic exchange between fissure microorganisms. Retention is one of the most critical properties of fissure sealants. This in vivo study is aimed at comparing and evaluating the clinical efficacy of resin and glass ionomer-based fissure sealants on first permanent molars with follow-ups at 6-, 12-, and 18-month intervals.

**Methods:**

A randomized split-mouth design clinical study was conducted after obtaining the ethical committee approval. A total of 50 patients, aged between 7 and 12 years, were randomized and enrolled in the study to perform a total of 200 sealant placements on all four caries-free and hypoplasia-free first permanent molars having deep fissures, which are susceptible to caries, were included in this study. The four permanent molars were divided into the following four groups: group A (control), B (Grandioseal, Voco, Germany), C (Smartseal & Loc, Detax Gmbh & Co, Germany), and D (Fuji triage capsule, GC, Belgium). The sealed molars were clinically evaluated at intervals of 6, 12, and 18 months to assess sealant retention, surface roughness, marginal coloration, and caries status through visual evaluation of the sealant by two evaluators.

**Results:**

Concerning retention, there were statistically significant differences between the sealants in terms of the survival of partial and fully retained sealants as well as in the survival of caries-free teeth. Two resin-based (Smartseal & Loc) and glass-ionomer cement (Fuji triage) sealants showed significantly similar performances in permanent molars for up to 18 months. In terms of retention, one of the resin-based (Grandioseal) sealants performed better as compared to the others and showed better caries prevention in deep fissures.

**Conclusion:**

It is concluded that both the sealants had comparable retention and caries-preventive effects in 7 to 12-year-old children and can be considered as suitable sealants for a period of at least 18 months in moderate caries risk patients.

## 1. Introduction

Fissure sealants are useful for preventing dental caries in fissures on the surface of permanent teeth in children [1]. The American Academy of Pediatric Dentistry (AAPD) stated that fissure sealants reduce caries by 76% [2]. Fissure sealant materials are generally classified according to their ingredients. There are polyacid-modified resin sealants (PRSs), resin-modified glass-ionomer sealants (RGSs), glass-ionomer sealants (GSs), and resin-based sealants (RSs) available in the market. RS includes monomers polymerized by light or chemical activators and are classified into four generations according to their polymerization. The first generation was polymerized by ultraviolet light while the second generation was chemically cured sealants or autopolymerizing RS. Light-polymerizing RS was the third generation while the fourth generation was the RS that included fluoride-releasing particles. GS is derived from the acid-base reaction between a polyacrylic acid solution and a fluoroaluminosilicate glass [3]. Although it has been declared that GS has low resistance to masticatory forces and its retention rates are lower than RS [4, 5], it has several advantages. The application of GS is easier than RS. It bonds the teeth with a chemical reaction and can be applied without pretreatment [2]. In addition, GS is not sensitive to moisture and enables adhesion and fluoride release. On the other hand, RS has no or minimal fluoride release. Markovic et al. reported that the long-term retention rate of GS is low; however, this material prevented caries formation in 65% of permanent molar fissures [6].

The clinical capability of the operator, the type of fissure sealant, and the compliance of children could influence the retention of these materials. When a meta-analysis studied the retention rates of fissure sealant materials with regard to the different materials and examination times, fluoride-releasing and light-polymerizing sealants displayed the best retention rates [7]. PGS and GS showed lower retention rates than RS [8]. However, it has been stated that with improvements in material technologies, high-viscosity glass-ionomer cements showed an improved retention rate as compared to resin-based sealants [9].

The null hypothesis is that sealants with high retention rates which have the capacity to stay in the mouth for a long time will be effective in preventing caries. The retention of resin fissure sealants is longer than glass-ionomer cements. However, there is still a lack of literature on the long-term clinical results of GS and RS. This controlled randomized clinical trial is aimed at analyzing the 18-month success of different types of sealants in vivo.

## 2. Material and Methods

The study protocol of this randomized, controlled, clinical trial was approved by the Ethics Committee of the Ege University (ethical code: 12-10.1/4). The aim of the study, its procedures, and its related risks were explained to the children and their parents before its commencement. Informed consent forms were signed by all the parents. The study was planned to cover all first permanent molar teeth, where one of them was left untreated, to serve as the control. The remaining three first permanent molars received different fissure sealant materials. The randomization of the applications per tooth was conducted using the envelope technique. Each tooth was allocated to a study group where all groups, including the control, contained an equal number of upper/lower/left/right first molars. The operators (IU, CG, and BK) selected the treatments that were already blindly allocated to a group from an envelope. The fissure sealants were applied by three authors, and follow-ups were conducted after the 6^th^, 12^th^, and 18^th^ months by two blind evaluators using the modified Ryge criteria [10].

The sample size required for each group was determined to be at least 48 teeth (*n* = 192 total restoration) using G-power software™ version 3.1.9.7 for Windows (Heinrich Heine, Universitat, Dusseldorf, Germany), for a power of 89% (*α* = 0.05, 1 − *β* = 0.885).

A total of 200 first permanent molars were included in the study. The study included 50 children aged between 7 and 12 years attending the pediatric dentistry clinic of the university, with 38 children being followed up at the end of 18 months. The oral hygiene status of the children was also recorded at the first visit as well as during the 6^th^, 12^th^, and 18^th^ months. Their oral hygiene status was categorized into three groups: poor, medium, and good.

The selection of the children was based on the following inclusion/exclusion criteria:

Inclusion criteria are as follows:

- Children aged between 7 and 12 years who were healthy, without any known history of systemic illness
- Children whose maxillary and mandibular first permanent molars have completely erupted with sound and intact fissures
- Children whose first permanent molars consist of deep fissures with 0 and 1 scores, according to ICDAS classification
- Children who had not received fluoride and/or fissure sealant application
- Children who may attend the clinic regularly for controls throughout the 18 months

Exclusion criteria are as follows:

- Children with special needs
- Uncooperative children
- Children with enamel hypoplasia, dental fluorosis, or suspected caries
- Children enrolled in any fluoridation program
- Children with bruxism or parafunctional habits
- Children with teeth that receive excess or no load due to malocclusion
- Children whose teeth have insufficient isolation and, thus, cannot be treated with the specified application technique

The teeth were randomly divided into the control or one of the three study groups using the envelope technique. All three first permanent molars of each patient were sealed in the same session by three authors (IU, CV, and BK). The study groups were as follows: group 1: control (no treatment), group 2: Grandioseal (Voco, Germany), group 3: Smartseal & Loc (Detax Gmbh & Co), and group 4: Fuji triage capsule (GC Europe, Belgium).

A probe was used to ensure the marginal seal of the fissure sealant. As a policy of the clinic, all children in the study and control groups received oral health education during their regular visits.

Design and application of fissure sealants

Four first permanent molars of each child were randomly designated for study and control groups. All tested materials were used according to the manufacturers' instructions.

Group 1: control

After polishing with pumice, no sealant application was carried out and the fissure was evaluated for discoloration and caries.

Group 2: Grandioseal resin fissure sealant

Phosphoric acid (37%) was applied to the fissures of the teeth for 30 seconds. The acid was removed with plenty of air-water sprays. All surfaces were dried. The fissure sealant was applied to the fissures of the tooth. It was light-cured with a light-emitting diode curing unit (3M, Elipar, USA) set at a standard power for 20 seconds. A probe was used to check the fissures in order to ensure the marginal seal between the sealant and the tooth surface. Finishing and polishing were completed during the same appointment.

Group 3: Smartseal & Loc resin fissure sealant

Phosphoric acid (37%) was applied to the fissures of the teeth for 30 seconds. The acid was removed with plenty of air-water sprays and dried with a cotton wool pellet for wet bonding. A thin layer of fissure sealant was applied to the fissures of the tooth. A light-emitting diode curing unit (3M, Elipar, USA) set at a standard power was applied for curing the sealant for 20 seconds. The marginal seal between the sealant and the tooth surface was checked. Finishing and polishing were performed during the same appointment.

Group 4: Fuji triage capsule fissure sealant

A GC cavity conditioner was applied for 10 seconds. The acid was rinsed with air-water spray and dried with a cotton pellet. The Fuji triage capsule was activated just before mixing and was used immediately. The tooth was isolated for 5-6 minutes to provide time for the setting of the glass-ionomer material. Finishing and polishing were performed during the same appointment using.

Evaluation procedure

The retention rate, marginal adaptation, surface roughness, staining, and visual evaluation of the fissure sealants were clinically evaluated using a dental explorer and mirror following the modified Ryge criteria in the study. All surfaces of the teeth included in the study were evaluated in terms of caries formation as well. As a preliminary study for this research, two experienced examiners (EE and FE) evaluated 15 patients with previously sealed fissures and 5 patients with no treatment on their first permanent molars (control group) for calibration and reached a consensus on the modified Ryge criteria. The examiners were unaware of the materials used. In cases of disagreement between the examiners, a mutual decision was reached through reevaluation and an agreement was achieved.

The examination results were categorized, according to the modified Ryge criteria, into three groups:

Retention criteria are as follows: complete retention—successful: 1, clinically acceptable: 2, and no retention—unsuccessful: 3. Marginal adaptation, surface roughness, surface staining, and visual evaluation criteria are as follows: successful: 1, acceptable: 2, and unsuccessful: 3. Oral hygiene status is as follows: good: 1, medium: 2, and poor: 3. Caries status (presence or absence) is as follows: caries: 1 and no caries: 2.

### 2.1. Statistical Analysis

The statistical analysis was conducted using the SPSS 18 (SPSS Inc, Chicago, USA), with the statistical significance set at *P* < 0.05. Descriptive statistics, Chi-square, and Kaplan-Meier tests were employed to evaluate the effect of oral hygiene on the retention of fissure sealants.

## 3. Results

A total of 50 children (28 girls and 22 boys) aged between 7 and 12 years (mean age: 8.18 ± 1.22), all of whom had four intact first permanent molars, were randomly enrolled in the study. The dft, dfs, and DMFT scores of the children are presented in Table 1.

### 3.1. Baseline

All the groups were successful in the baseline evaluation. There was no significant difference between the groups in terms of retention, marginal adaptation, surface roughness, and visual evaluation (*P* = 1). There was also no significant difference between the groups in terms of oral hygiene (*P* = 0.315).

### 3.2. 6^th^ Month

There was no significant difference between the groups in terms of retention, marginal adaptation, surface roughness, and visual evaluation (*P* = 0.476, 0.069, 0.069, and 0.35, respectively). There was also no significant difference between their marginal coloration and caries formation (*P* = 0.27 and 0.65, respectively).

### 3.3. 12^th^ Month

The Grandioseal sealant had better retention rates than the other groups, but there was no significant difference between the groups in terms of retention, marginal coloration, and caries formation (*P* = 0.052, 0.319, and 0.376, respectively).

There was a significant difference between the groups in terms of marginal adaptation, surface roughness, and visual evaluation (*P* = 0.013, 0.004, and 0.001, respectively). The Grandioseal sealant performed better than the other groups.

### 3.4. 18^th^ Month

There was a significant difference between the groups in terms of retention, visual evaluation, and caries formation (*P* = 0.046, 0.007, and 0.006, respectively) where the Grandioseal sealant performed better than the other groups. The control group had higher caries values than the others.

There was no significant difference between the groups in terms of marginal adaptation, surface roughness, and marginal coloration (*P* = 0.110, 0.256, and 0.798, respectively) (Table 2).

## 4. Discussion

A wide variety of materials are used as fissure sealants. However, they can be classified into two primary groups—RS and GS [11]. Although RSs are commonly preferred and used due to their gratifying retention rates, their placement is technically sensitive because of the hydrophobic Bis-GMA. New smart resin materials provide wet bonding efficiency to combat this disadvantage. On the other hand, clinically, GS has the highest tolerance to moisture. Although these materials are insufficiently retained and have low wear resistances [5], the release of fluoride and adhesion to the tooth surface are among the important features of GS. It is important to note that the primary aim of fissure sealing is the protection of healthy fissures; therefore, the effectiveness of fissure sealants is the prevention of the occurrence of a cavitated lesion, and its surrogate endpoint may be the survival of the fissure sealant.

There are several reports on the survival of currently available fissure sealants in the market. Ulusu et al. reported that, after 6 months, 47% of RSs were successful, with only 11.9% of these materials missing. However, 45.7% of GSs were successful, and 24.5% of these materials were missing in the same study [12]. Bechir et al. declared that the retention ability of GS was lower than that of RS in a one-year clinical study [9]. Markovic et al. reported that 69% of GSs were successful after 1 year [6]. Alkhodairi et al. evaluated the retention of RS and GS to conclude that the retention of RS was 83.3% while that of GS was 63.3% after 3 months. They also found that 60% of the resin sealant and 55% of the glass-ionomer sealant were present after 6 months. There was a statistically significant difference between the two groups [5]. The retention of resin-based dental materials, such as sealants, composites, and luting cements, has been affected by both environmental factors and application procedures. The loss of fissure sealants may cause enamel defects similar to the ones observed in the debonding of orthodontic brackets [13]. Therefore, early loss of resin fissure sealants should be closely evaluated and retreated as soon as possible.

Cabral et al. stated that the retention rate of resin-based sealants was higher than glass-ionomer sealants [4]. Grassia et al., Ugur and Hande, Alsabek et al., and Fragelli et al. reported high complete retention rates for resin-based fissure sealants in their studies [13–16]. It was reported that the retention rate of resin-based fissure sealants was as high as 94.8% in the study by Ugur and Hande after one year [14].

The success of a fissure sealant depends not on its retention but on its caries-preventive effect. It is thought that the anticaries effect of glass ionomer-based sealants could be related to the fact that they remain in the deepest parts of the fissures [17]. Also, the fluoride-releasing ability of the glass ionomers could impact the anticaries effect [18]. When the caries-preventive effect of glass ionomer-based fissure sealants was compared to that of resin-based sealants, no significant difference was found at 24-, 36-, and 48-month intervals [19]. However, a significant increase in the anticaries effect was found in favor of glass-ionomer sealants at the 60^th^ month evaluation. Haznedaroglu et al. stated that the anticaries effect of glass ionomer-based fissure sealants was higher than resin-based sealants, although the retention rate of the former was significantly lower than the latter [20]. The American Dental Association (ADA) and the American Academy of Pediatric Dentistry (AAPD) have not yet reported any results on which of the two sealants is better due to the low quality of available findings [1, 2]. Glass ionomer-based fissure sealants could render better results in caries prevention and marginal staining as compared to resin-based sealants on teeth that have not completely erupted [21]. However, there was no significant difference in retention between the two sealant materials in partially erupted teeth. Thus, it was concluded that glass ionomer-based fissure sealants could be a better material than resin-based fissure sealants for sealing partially erupted teeth, because of insufficient isolation.

No marginal discoloration was recorded on teeth sealed with glass-ionomer fissure sealants; however, minor (6%) marginal discoloration was noted for teeth sealed with a resin fissure sealant. At the same time, 2% of the teeth sealed with glass ionomer-based sealant improved caries while none of the teeth with resin-based sealant improved caries in the one-year clinical study [11]. However, there was no statistically significant difference between RS and GS in terms of retention rate, anticaries effect, and marginal discoloration in the study.

The success of the resin-based fissure sealant is closely related to the operator, and the lack of good outcome could be a result of the inability of the dentist and the placement technique [22]. Alkhodairi et al. stated that the GS has insufficient retention but is less technique sensitive [5]. Sealing during tooth eruption presents a particular challenge owing to the difficulty in isolating the tooth. Glass ionomers may be a better material for sealing partially erupted molars. The findings of this study conclude that fissure sealants from different materials are effective in caries prevention. Further improvements in the availability of sealant materials may improve the retention rates, and the success could then be attributed to the retention of sealants.

Due to the limited number of sealants applied in this study, the operator effect could not be reported. In this study, lower survival rates could have been reached if the follow-ups had been extended for a longer period.

## 5. Conclusions

In this study, glass ionomer-based and wet-bonding resin-based fissure sealants significantly exhibited the same clinical outcomes over the observation period of 18 months. Consequently, the null hypothesis formulated at the beginning of the present study was rejected. When the clinical results of the findings of this study were examined from a different perspective, it was found to be crucial. Encapsulated glass-ionomer cement sealant features are important for clinical practice in pediatric dentistry. It has the advantage of chemical adhesion of the glass ionomers to tooth structures without the need for a light cure and entails a simple application technique. Observationally, the use of a glass ionomer-based sealants takes lesser time than composite sealants. Also, the use of glass-ionomer cement is preferred over composite materials because of their biocompatibility and, especially, for the fluoride release/recharge from the glass component.

## Figures and Tables

**Table 1:** Caries status of children in the study.

	Age mean ± SD	dft mean ± SD	dfs mean ± SD	DMFT mean ± SD
Boys	8.42 ± 1.33	3.42 ± 2.75	4.71 ± 4.10	0.06 ± 0.25
Girls	7.79 ± 0.91	2.00 ± 2.47	3.21 ± 4.32	0.11 ± 0.31
Total	8.18 ± 1.22	2.88 ± 2.71	4.14 ± 4.21	0.08 ± 0.27

**(a):** 

		Grandioseal	Smartseal	Fuji triage	*P* value
*Retention loss*					
Baseline	Successful	50 (100%)	50 (100%)	50 (100%)	1.00
	Acceptable	-	-	-	
	Unsuccessful	-	-	-	
6-month	Successful	41 (95.3%)	37 (86.0%)	38 (88.4%)	0.476
	Acceptable	0 (.0%)	3 (7.0%)	3 (7.0%)	
	Unsuccessful	2 (4.7%)	3 (7.0%)	2 (4.6%)	
12-month	Successful	25 (65.8%)	13 (34.2%)	16 (42.1%)	0.052
	Acceptable	8 (21.1%)	11 (29%)	9 (23.7%)	
	Unsuccessful	5 (13.1%)	14 (36.8%)	13 (34.2%)	
18-month	Successful	17 (51.6%)	8 (24.2%)	6 (18.2%)	0.046
	Acceptable	8 (24.2%)	12 (36.4%)	13 (33.3%)	
	Unsuccessful	8 (24.2%)	13 (39.4%)	14 (42.5%)	

*Marginal adaptation*					
Baseline	Sound	50 (100%)	50 (100%)	50 (100%)	1.00
	Acceptable	-	-	-	
	Missing	-	-	-	
6-month	Sound	41 (95.3%)	36 (83.7)	41 (95.3%)	0.069
	Acceptable	0 (.0%)	4 (9.3%)	0 (.0)	
	Missing	2 (4.7%)	3 (7.0%)	2 (4.7%)	
12-month	Sound	29 (76.3%)	15 (39.5%)	21 (55.3%)	0.013
	Acceptable	4 (10.5%)	10 (26.3%)	4 (10.5%)	
	Missing	5 (13.2%)	13 (34.2%)	13 (34.2%)	
18-month	Sound	21 (63.7%)	11 (33.3%)	14 (42.4%)	0.110
	Acceptable	4 (12.1%)	9 (27.3%)	5 (15.2%)	
	Missing	8 (24.2%)	13 (39.4%)	14 (42.4%)	

*Surface roughness*					
Baseline	Successful	50 (100%)	50 (100%)	50 (100%)	1.00
	Acceptable	-	-	-	
	Unsuccessful	-	-	-	
6-month	Successful	41 (95.3%)	36 (83.7%)	41 (95.3%)	0.069
	Acceptable	0 (.0%)	4 (9.3%)	0 (.0%)	
	Unsuccessful	2 (4.7%)	3 (7.0%)	2 (4.7%)	
12-month	Successful	29 (76.3%)	15 (39.5%)	22 (57.9%)	0.004
	Acceptable	4 (10.5%)	10 (26.3%)	2 (5.3%)	
	Unsuccessful	5 (13.2%)	13 (43.2%)	14 (36.8%)	
18-month	Successful	18 (54.5%)	12 (36.4%)	16 (48.5%)	0.256
	Acceptable	7 (21.3%)	8 (24.2%)	3 (9.1%)	
	Unsuccessful	8 (24.2%)	13 (39.4%)	14 (42.4%)	
*Visual evaluation*					
Baseline	Successful	50 (100%)	50 (100%)	50 (100%)	1.00
	Acceptable	-	-	-	
	Unsuccessful	-	-	-	
6-month	Successful	41 (95.3%)	38 (88.4%)	41 (95.3%)	0.350
	Acceptable	0 (.0%)	2 (4.6%)	0 (.0)	
	Unsuccessful	2 (4.7%)	3 (7.0%)	2 (4.7%)	
12-month	Successful	32 (83.8%)	16 (42.1%)	22 (57.9%)	0.001
	Acceptable	1 (2.7%)	9 (23.7%)	2 (5.3%)	
	Unsuccessful	5 (13.5%)	13 (34.2%)	14 (36.8%)	
18-month	Successful	24 (72%)	11 (33.3%)	15 (45.5%)	0.044
	Acceptable	1 (3.0%)	9 (27.3%)	4 (12.1%)	
	Unsuccessful	8 (24%)	13 (39.4%)	14 (42.4%)	

**(b):** 

		Control	Grandioseal	Smartseal	Fuji triage	*P* value
*Marginal coloration*						
Baseline	Successful	47 (94.0%)	50 (100%)	48 (96.0%)	49 (98.0%)	0.33
	Acceptable	3 (6.0%)	0 (.0%)	1 (2.0%)	1 (2.0%)	
	Unsuccessful	0 (.0%)	0 (.0%)	1 (.2.0%)	0 (.0%)	
6-month	Successful	40 (93.0%)	43 (100.0%)	42 (97.7%)	42 (97.7%)	0.27
	Acceptable	3 (7.0%)	0 (.0%)	1 (2.3%)	1 (2.3%)	
	Unsuccessful	-	-	-	-	
12-month	Successful	31 (81.6%)	32 (84.2%)	29 (76.3%)	28 (73.7%)	0.31
	Acceptable	5 (13.2%)	3 (7.9%)	5 (13.2%)	2 (5.3%)	
	Unsuccessful	2 (5.3%)	3 (7.9%)	4 (10.5%)	8 (21.2%)	
18-month	Successful	24 (72.7%)	24 (72.7%)	22 (66.7%)	22 (66.7%)	0.79
	Acceptable	6 (18.2%)	5 (15.2%)	7 (21.2%)	4 (12.1%)	
	Unsuccessful	3 (9.1%)	4 (12.1%)	4 (12.1%)	7 (21.2%)	
*Caries status*						
Baseline	No caries	50 (100%)	50 (100%)	50 (100%)	50 (100%)	
	Caries	-	-	-	-	
6-month	No caries	40 (93%)	41 (95.3%)	42 (97.7%)	42 (97.7%)	0.65
	Caries	3 (7.0)	2 (4.7%)	1 (2.3%)	1 (2.3%)	
12-month	No caries	34 (89.50%)	36 (94.7%)	37 (97.4%)	1 (97.3)	0.37
	Caries	4 (10.5%)	2 (5.3%)	1 (2.6%)	1 (2.7%)	
18-month	No caries	26 (74.3%)	29 (90.6%)	32 (97.0%)	32 (97.0%)	0.37
	Caries	9 (25.7%)	3 (9.4%)	1 (3.0%)	1 (3.0%)	

## Data Availability

Derived data supporting the findings of this study are available from the corresponding author on request.
